The article "Design of a Fuzzy Algorithm-Based Evaluation System for the Effectiveness of International Online Chinese Listening and Speaking Teaching" was retracted in 2023. Reasons: signs of a paper mill; suspected computer-generated content; unreliable results or conclusions; lack of ethics approval or compliance.

# Design of a Fuzzy Algorithm-Based Evaluation System for the Effectiveness of International Online Chinese Listening and Speaking Teaching

**DOI:** 10.1155/2022/8135282

**Published:** 2022-08-22

**Authors:** Dong Ge, Tianyu Wang, Chunhong Qi, Shan He

**Affiliations:** ^1^Global Innovation Academy, Siam University, 38 Petchkasem Road, Phasi Charoen, Bang Wa, Bangkok 10160, Thailand; ^2^College of International Chinese Language Education, Yunnan Normal University, Juxian Street, Chenggong District, Kunming, Yunnan Province 650500, China

## Abstract

With the increasing popularity of online foreign language teaching and learning practice, learners and teachers have developed a high demand for evaluation of teaching effectiveness. When we focus discussion on international Chinese teaching, which has been developed for a relatively short time and not experienced enough, online teaching effectiveness evaluation has become an important obstacle to the development of teaching. This paper introduces a hybrid technique based on fuzzy evaluation method, for determining and suggesting possible types of errors in international Chinese online listening and speaking instruction and giving suggestions for improvement. The system can help learners to identify and determine the types of errors in Chinese listening and speaking learning in a timely manner and make a more objective and comprehensive evaluation of learning performance; at the same time, it helps teachers to trace the effectiveness of teaching design and implementation in a targeted manner and make corresponding scientific decisions. This hybrid technology combines existing language teaching evaluation models, takes advantage of data from online education, and creates corresponding criteria through machine learning fuzzy algorithms and large data sample training, combined with the theory of effective teaching evaluation, which is beneficial for all participants of online Chinese listening and speaking teaching to improve their learning effectiveness.

## 1. Introduction

With the development and popularity of information and network technologies, online learning, which can meet learners' individual needs to a greater extent, has attracted more and more learners because it creates a rich and diverse educational environment that allows learners to access information, experience learning, interact with peers and teachers, and participate in campus-wide co-curricular programs [1], and foreign language learners around the world occupy a high percentage of the online learner population [2]. Since the global outbreak of the novel coronavirus in 2020, online learning has gradually become an inevitable choice for foreign language teaching and learning, not only for international learners around the world, but also for local learners in countries and regions experimenting with outbreak control. The increasing complexity of the online learning environment poses a great challenge to the assessment of their learning experience [3], and the evaluation of teaching effectiveness has become an important part of it. However, compared to traditional offline foreign language teaching evaluation methods, the virtual environment of online teaching, technological limitations, learners' psychology of distance learning, and individualized learning needs all have a non-negligible impact on the achievement of teaching effectiveness.

Chinese is a fast-growing foreign language learning field in the world in recent years, and the number of learners is increasing rapidly. However, compared with English education and other foreign language teaching fields that have been developed for a long time, the online Chinese language learning community is still “a relatively underestimated group of learners” [4], and there is not enough research on international online Chinese language teaching. At the same time, since Chinese is recognized as a difficult language to learn worldwide, it has unique language system characteristics (pronunciation, glyph, and meaning of character are constructed as a whole); the lack of face-to-face interaction and the “distance” of online teaching may pose additional barriers to learning Chinese, especially the tones and characters in the Chinese language system [5, 6]. At the same time, the understanding of Chinese listening and speaking is very dependent on the context, on account of there are a large number of homophones and near words in Chinese. However, the evaluation system based on the effectiveness of online Chinese teaching has not been fully constructed, and the evaluation methods that can provide reference for teachers and learners still rely too much on the traditional offline teaching scenes. Based on these challenges, the use of scientific and effective ways to rationalize the effectiveness of teaching and learning has become an important and meaningful issue in the development of international online Chinese language teaching.

The authors of this paper have been teaching Chinese internationally for a long time and have accumulated a certain amount of conversational bias corpus of primary, intermediate, and advanced (based on International Chinese Proficiency Test—HSK grading standards) Chinese learners in listening and speaking classes and have preliminary analyzed and discussed these biases and the reasons for them [7]. Since 2020, three teachers in the research team have been teaching online Chinese courses to international students through online teaching and have accumulated some experience on the issue of evaluating the effectiveness of online listening and speaking classes.

Before conducting this study, we had tried to help improve the effectiveness of online international Chinese listening and speaking classes by conducting one-on-one interviews, focus group discussions, questionnaires, and brainstorming with some instructors and learners with more focused feedback on learning problems, but the results were still very ineffective. Through the exchange with IT experts, we realized that the evaluation environment of online teaching is quite different from traditional offline teaching, so the basis of evaluation must return to online teaching itself, to this virtual teaching time and space constructed by technology. A new perspective on the evaluation logic and model from a technological perspective became the starting point of our new round of research.

The research objectives of this paper mainly include the following: based on the current status and network conditions of international Chinese listening and speaking class teaching, (1) designing an evaluation model of online Chinese listening and speaking teaching effectiveness based on machine learning and fuzzy algorithm; (2) applying experiments to verify the feasibility and effectiveness of the model; and (3) discussing the factors affecting the effectiveness of online Chinese listening and speaking teaching and its mechanism of action from the technical perspective.

## 2. Design Framework of FOCLSTEES

### 2.1. Fuzzy Logic of FOCLSTEES

Second language learning is closely related to the language environment, and since the new millennium, the use of information technology in teaching and learning has brought new opportunities and challenges to the perceptions of learners and teachers [8]. For listening and speaking instruction, well-designed and functioning online learning may be beneficial for learners [9]. However, the high interaction distance between teachers and students that exists in online teaching and learning environments can also create obstacles to the creation of a language environment, and the model of one teacher dealing with multiple students at the same time (one-to-many) in most classroom settings may also create problems for the teacher's immediate learning feedback to students and its accuracy, to the detriment of the three types of interactions that educators should provide in distance education: learner-content; learner-instructor, and learner-learner [10–12] are generated. An innovative study conducted by Charles Dziuban and Patsy Moskal reviewed student evaluation of instruction (SEI) and its factors in online learning and found through an empirical study with a large sample (*n* = 1,124,979) that learners faced with either online, blended, or face-to-face course modalities; there were no significant differences in the dimensions of their course assessment experience [1]; and the strongest predictor of course instructional success was still academic achievement [13]. The authors also caution that it may be useful to consider new instructional assessment protocols that are not summative and post hoc, but rather those that are more reflective and interactive. With this in mind, our study places the starting point for evaluating the effectiveness of international online Chinese listening and speaking instruction in terms of learners' academic achievement, i.e., the extent to which they have acquired and mastered the knowledge and skills provided in the course instruction, and achieved the set goal of instructional design. The fuzzy logic of FOCLSTEES is to rationally present and analyze uncertain states of information representation by mimicking a face-to-face instructional environment and teacher-student thinking. The starting point of FOCLSTEES design is a rational mathematical model that processes teaching phenomena and events through fuzzy algorithms in order to eliminate fuzzy judgment logic.

Based on the context word embedding pretraining model (PTM) [14], FOCLSTEES can embed, organize, and subdivide the teaching contents of online Chinese listening and speaking courses according to the basic units of the Chinese language (words and sentences). These contents will judge whether learners need to embed context dynamics in the learning process according to the context or semantics, which helps teachers decide whether to adjust the teaching contents. We select the mask language model (MLM)/self-coding language model (context embedding module) for embedding [15], and the algorithm is as follows:

(1) $$\begin{array}{c} L_{MLM}=-\underset{\hat{x}\in m\left(x\right)}{\sum }\log p\left(\left.\hat{x}\right|x_{\bar{m}\left(\text{x}\right)}\right). \end{array}$$

In addition, FOCLSTEES is able to fuzzify the signal input (fuzzy control module) [16] for the facial expression feature signal, mouth image signal, and speech waveform signal that appear during the learners' online Chinese listening and speaking learning process, by accessing the evaluation database and corpus to the system according to the following flow (shown in Figure 1). The input signal E is a deterministic signal, which is first converted into a fuzzy signal $\underset{\sim }{E}$, and then combined with Chinese fuzzy concepts to configure control rules (rules from roundtable discussions with expert groups and literature study) to generate a new fuzzy relationship: $R=\underset{\sim }{E}\times \underset{\sim }{U}$, where *R* is the Chinese heard fuzzy control rule, and when the actual input is $\underset{\sim }{e}$, the fuzzy output is $\underset{\sim }{u}=\underset{\sim }{e}\circ R$, which is output after defuzzification (or called defuzzification) to complete the fuzzy controller control function.

### 2.2. Functional Design of FOCLSTEES

Based on the research team's long-term experience in offline Chinese teaching, we designed functional modules for FOCLSTEES, including three temporal state modules for pre-class preview, in-class learning, and post-class review, and three user-dimension modules for teachers, students, and administrators. The idea of module design comes from the current standard process of international Chinese teaching and the division standard of user groups in the school management system. In addition, in order to meet the needs of online teaching, the system also integrates the functions of live listening and hearing, video and digital playback, and material downloading and sets up online plug-ins to improve the system functions, such as note taking plug-in [17], quiz online [18], online textbook finger reading plug-in, classroom collaboration discussion plug-in [19], online quiz plug-in, classroom voting plug-in, and answer collection plug-in. In addition, the system also provides user personalized editing, personalized learning plan and progress design, animated presentation of lecture contents, spoken pronunciation and oral correction based on Chinese corpus (including playback, replay and recorded correction), learning report generation, and learning strategy suggestion.

### 2.3. Intelligent Extension of FOCLSTEES

In the traditional face-to-face foreign language teaching mode, a teacher faces multiple students at the same time, it makes teachers and their instructional design difficult to meet the individual needs of learners, and the teaching implementation follows the “T2S” (teacher-to-student) design logic [20, 21]; however, FOCLSTEES, thanks to the intervention of big data, machine learning, and information technology assistance, is able to continuously record and analyze the real-time data of teacher and student behavior (see Figure 2). With the intervention of big data, machine learning, and information technology, FOCLSTEES is able to record and analyze real-time data of teachers' and students' classroom behaviors, thus creating the possibility for the “S2T” (student-to-teacher) design model (see Figure 2).

The “S2T” model can help learners set personalized learning goals, choose appropriate learning strategies and problem solutions, develop their independent learning behaviors and abilities, carry out interaction and collaborative learning among learners, and obtain different forms of learning based on real-time automatic assessment and monitoring functions. It also provides teachers with the most direct and accurate decision-making advice for effective teaching. With the in-depth research of FOCLSTEES “S2T” model, according to the development of the industry, S2T2S, T2S2M, S2T2R, S2R, S2E, S2T2M, S2E2R, and other models will be deduced and evolved.

## 3. Principle of Comprehensive Evaluation and Data Configuration of FOCLSTEES

### 3.1. Comprehensive Validity Evaluation of FOCLSTEES

Summative evaluation and process evaluation are two common perspectives in international Chinese teaching effectiveness evaluation, but the data collected by these two evaluation models are either cross-sectional data based on a certain point in time or their comprehensive data sets. With the full amount of online teaching data recorded, FOCLSTEES can provide comprehensive and diverse assessment strategies, based on the diversity, authenticity, and speed of assessment design. The system can help learners effectively improve their learning participation through the “s2t” mode. In addition, based on the various modules and plug-ins provided by the system, FOCLSTEES can manage the whole process of students' online learning indicators, including the supervision of the whole process of online submission, grading, review and data storage, sample extraction learning, and fuzzy feature classification, providing data for the next stage of computer grading and human intervention. This provides data support for the next stage of computerized scoring and human intervention.

FOCLSTEES combines the standard pronunciation of the online Chinese listening and speaking course corpus with the steps of sound and image data collection, contextual embedding, data filtering, fuzzy processing, normalization, fuzzy feature extraction, etc., which are calculated by fuzzy subsets and fuzzy matrices, and finally combined with the database of manual evaluation opinions of course experts collected in the early stage to identify error types and provide the final comprehensive evaluation and improvement suggestions (as shown in Table 1).

The algorithm for the comprehensive evaluation is as follows:

(2) $$\begin{array}{c} \text{B}=\left(\begin{array}{c} {\text{A}}_{1}\\ {\text{A}}_{2}\\ {\text{A}}_{3}\\ \vdots \\ {\text{A}}_{m} \end{array}\right)\left(\begin{array}{ccccc} {\text{A}}_{11} & {\text{A}}_{21} & {\text{A}}_{31} & \cdots & {\text{A}}_{m1}\\ {\text{A}}_{12} & {\text{A}}_{22} & {\text{A}}_{32} & \cdots & {\text{A}}_{m2}\\ {\text{A}}_{13} & {\text{A}}_{23} & {\text{A}}_{33} & \cdots & {\text{A}}_{m3}\\ \vdots & \vdots & \vdots & \cdots & \vdots \\ {\text{A}}_{1j} & {\text{A}}_{2k} & {\text{A}}_{3l} & \cdots & {\text{A}}_{mn} \end{array}\right)={\text{A}}_{1}\cdot \left({\text{A}}_{11}+{\text{A}}_{12}+{\text{A}}_{13}+\cdots {\text{A}}_{1j}\right)+{\text{A}}_{2}\cdot \left({\text{A}}_{21}+{\text{A}}_{22}+{\text{A}}_{23}+\cdots {\text{A}}_{2k}\right)+\cdots {\text{A}}_{m}\cdot \left({\text{A}}_{m1}+{\text{A}}_{m2}+{\text{A}}_{m3}+\cdots {\text{A}}_{mn}\right). \end{array}$$

The Lever1 Indicators is “A1-Am,” and the Lever2 Indicators is “Amn” of the corresponding Level1 Indicators. According to the above formula, we can calculate the corresponding comprehensive examination judgment table “B,” and according to the above formula, we can calculate the corresponding comprehensive examination judgment table “B”, and can flexibly configure it with the actual teaching situation.

Finally, the comprehensive validity evaluation does not mean that it is the final evaluation, and it can then be considered further improved after adding expert information to correct the bias [22, 23] for use in the subsequent teaching process.

We first used the corpus data accumulated in the team's previous research to conduct application tests to ensure that the system could achieve smooth operation; next, we invited five teaching experts outside the team (whose personal experiences include teaching Chinese to international students for more than 10 years and teaching online Chinese listening and speaking since 2020) to evaluate FOCLSTEES' judgment of the types of Chinese listening and speaking learning errors, and the accuracy of the commentary results was evaluated. The experts will make necessary amendments and supplements to the results of the system identification. The contents after the amendments and supplements will be discussed by the research team and the experts at the round table meeting. The team will enter the agreed supplements into the system information base as the basis for the next round of testing. The judgments of FOCLSTEES come from expert were evaluated according to the scoring criteria of the 5-point Likert scale ((1) completely inaccurate; (2) partially inaccurate; (3) basically accurate; (4) mostly accurate; and (5) completely accurate), and then the Kendall's harmony coefficient of the evaluation results of the three experts was calculated, and the results showed that W^a^ = .825, *p* ≤ 0.001, and it indicates that the expert evaluations have high consistency and FOCLSTEES runs well for error type identification and commenting.

### 3.2. Validity Feedback and Fuzzy Control of FOCLSTEES

FOCLSTEES further investigates the close relationship between assessment, feedback, and effective teaching. We found that the comprehensive assessment results after fuzzy identification and after data processing, continue to enhance the feedback to the system, which can again be used as neurons for machine learning and repeatedly input into the “hidden layer” iterative computation (neural network), which can repeatedly optimize the student learning results.

After many iterations of teaching and learning processes, the triggering of new fuzzy data generates a new *R*^(*l* + 1)^, and this new comprehensive evaluation data (CED) can be reverse resolved to the various types of metadata that triggered it (see Figure 3 for details), and this batch of metadata, which can be used as a supervised sample for the next iteration, participates in the fuzzy learning of the neural net.

The feedback algorithm process for processing and continuing enhancement of the fuzzy data after the integrated evaluation [24] is as follows:

Step 1: Select the classification number*c*(2 ≤ *c* ≤ *n*), input the fuzzy data after the previous comprehensive evaluation, find its corresponding first and second level metadata, and process it and input it to the “hidden layer”; the new generation fuzzy classification matrix is*R*^(0)^ = (*r*_*ij*_^(0)^)_*c*×*n*_ ∈ *M*_*fc*_, which can be iterated as many times as needed: *l* = 0, 1, 2, ⋯

Step 2: For *R*^(*l*)^, calculate the cluster center matrix *V*^(*l*)^ = (v_1_^(*l*)^, v_1_^(*l*)^, ⋯, v_*c*_^(*l*)^); here, *V*_*i*_^(*l*)^, which can be calculated as follows:

(3) $$\begin{array}{c} {V_{i}}^{\left(l\right)}=\frac{\sum_{k=1}^{n}{\left(r_{ik}^{\left(l\right)}\right)}^{q}u_{k}}{\sum_{k=1}^{n}{\left(r_{ik}^{\left(l\right)}\right)}^{q}},\left(i=1,2,\cdots ,c\right). \end{array}$$

Step 3: Correct the fuzzy clustering matrix *R*^(*l*)^, taking

(4) $$\begin{array}{c} {r_{ik}}^{\left(l+1\right)}={\left[\overset{c}{\underset{j=1}{\sum }}{\left(\frac{\left\|u_{k}-V_{i}^{\left(\text{l}\right)}\right\|}{\left\|u_{k}-V_{j}^{\left(\text{l}\right)}\right\|}\right)}^{2/q-1}\right]}^{-1},\left(k=1,2,\cdots ,c\right). \end{array}$$

Step 4: Compare *R*^(*l*)^ with *R*^(*l* + 1)^, compare and image showing the difference; if FOCLSTEES has new data update, *l* = *l* + 1, go back to Step 3, go to the next iteration, and repeat

In general, the fuzzy clustering matrices *R*^(*l* + 1)^ and *V*^(*l*)^ obtained by applying the above algorithm are locally optimal solutions with respect to the number of classifiers *c*, the initial fuzzy clustering matrices *R*^(0)^ and *ε*, and the parameters *q*.

By recruiting volunteers, we analyzed the trial experience of 10 learners each at the beginner, intermediate, and advanced levels. Due to the small number of learners in a single group, the use of *t*-tests could not fully account for changes in learning effectiveness and whether they differed significantly. We used one-on-one interviews with a combination of structured and open-ended questions to understand their perceptions of use. In the structured section, 86% of trialists reported that FOCLSTEES had significant reinforcement for learning (91% for beginners, 88% for intermediate, and 79% for advanced), but there were differences in the ratings of trialists at different levels, with learners at higher levels rating it lower. The experience of the previous related study [7] is consistent with this result; as the level of Chinese learning increases, the content of students' conversational correction is weighted from grammar, vocabulary, and phonology in descending order at the elementary level; vocabulary, grammar, and phonology at the intermediate level; and vocabulary, phonology, and grammar at the advanced level. In particular, there are a large number of near-synonyms and synonyms in the Chinese language system, and there are many changes in the language usage scenarios, which make machine learning and analysis difficult; in the unstructured open interview part, the trialers' experience also provided us with many useful ideas for future improvement of the system. “You know learning Chinese is really a painful thing, especially those vocal tones with subtle differences, and this system has definitely brought a lot of convenience to our Chinese listening and learning, but obviously it can do better in the future, and I'm looking forward to it giving more suggestions on the use of near-sense words” (20 years old, female, beginner); “I think using this system to help learn Chinese listening and speaking is efficient, it tells me a lot of mistakes that occur and I can recognize them immediately and fix them, which definitely saves time, both the student's and the teacher's. But I think it could also become smarter and tell us more about the use of authentic Chinese usage” (18 years old, male, advanced). The trial participants' evaluations gave hints that FOCLSTEES needs further refinement and improvement in handling error identification and evaluation of listening and learning for higher level learners.

## 4. Conclusion

Based on the experience of learners with different Chinese proficiency, the research team found FOCLSTEES helps improve the effectiveness of international online Chinese listening and speaking teaching, helps learners find and correct their mistakes in time, helps teachers adjust their teaching strategies and improve their teaching design, and puts the teaching process into a virtuous circle spiral. Although our exploration is still in a preliminary state, it should be recognized that the S2T (student-teacher) model proposed by the system is an effective exploration to improve the effectiveness of online Chinese teaching. In the preliminary study stage, it builds a personalized learning development idea after creating data between online Chinese listening and speaking instructors and students, realizes an online digital bridge between schools and students, and explores an effective way to improve the innovation ability and competitiveness of online education technology. One thing we can foresee is that, in the era of rapid development of information technology in distance education, the number of learners learning Chinese with the help of the Internet will continue to increase. The use of machine learning and fuzzy algorithms to provide real-time intelligent quantitative analysis for teaching evaluation, combined with the strategic use of expert manual assessment databases, is a useful reflection and experiment for online language teaching evaluation. In addition, when other online course teaching and online course data conditions are available and further explore S2T2S, T2S2M, S2T2R, S2R, S2E, S2T2M, S2E2R, and other models, there is no doubt that we can further work together to jointly promote the development of the online education industry. It should be said that FOCLSTEES technology can provide a new perspective for online Chinese listening and learning evaluation and also provide computational ideas for teaching evaluation of other online courses.

## Figures and Tables

**Figure 1:** Fuzzy control flow of international Chinese listening and speaking teaching.

**Figure 2:** FOCLSTEES S2T Mode. Notes: S (student), T (teacher), R (research), E (experiment), M (management), and 2 (to).

**Figure 3:** Reverse parsing to CED to the various types of metadata *R*^(*l*)^ schematic.

**Table 1:** Examples of Chinese listening and learning error types and FOCLSTEES comments.

Error type	Example of error	FOCLSTEES comments
Inaccurate intonation	Wǒ jīn tiān zhōng wǔ chī le [jiāo zi] (I had dumplings this noon)	There may be a tone error in this sentence [jiǎo zi] Please confirm the tones and try again
Mispronunciation of consonants	Wǒ zuó tiān [qì] le bó wù guǎn (I went to the museum yesterday)	There may be a mispronunciation of the consonant in this sentence [qù]. Please confirm the correct pronunciation of the consonant and try again
Polyphone pronunciation error	Wǒ fēi cháng xǐ huān zhè bù diàn yǐng zhōng de nán zhǔ [jiǎo] (I like the leading man in this movie very much)	There are polyphonic characters [jiǎo and jué] in this sentence. Please confirm the correct pronunciation of this word, and then try again. Polyphonic characters in Chinese characters will choose different pronunciation according to the context
Misordering of words	Mā ma ràng wǒ hē shuǐ yī bēi.(mother let me have a glass of water.)	This sentence may have been structured in the wrong Order; the quantifiers should be placed before the nouns. Please proofread the sentence to make sure that each part of the sentence is in the correct order.
Wrong use of verbs	Wǒ huì bāng máng tóng xué wán chéng zhè gè rèn wù (I will help my classmates complete this task)	There may be a mistake in the verb in this sentence, perhaps a confusion between [bāng zhù] and [bāng máng]. [bāng zhù] can be followed by an object, but [bāng máng] is not. Please proofread the sentence to make sure that the verbs are used in the correct way

## Data Availability

The data that support the findings of this study are available from the corresponding author upon reasonable request.
